The article "Accuracy of UWB Path Loss-Based Localization of Wireless Capsule Endoscopy" was published in 2023. Journal: J Healthc Eng.

# Accuracy of UWB Path Loss-Based Localization of Wireless Capsule Endoscopy

**DOI:** 10.1155/2023/3156013

**Published:** 2023-06-13

**Authors:** Umma Hany, Lutfa Akter

**Affiliations:** ^1^Department of Electrical and Electronic Engineering, Ahsanullah University of Science and Technology, Dhaka, Bangladesh; ^2^Department of Electrical and Electronic Engineering, Bangladesh University of Engineering and Technology, Dhaka, Bangladesh

## Abstract

Wireless capsule endoscopy (WCE) is used to diagnose lesions in the gastrointestinal (GI) tract. The physicians require to know the exact position of the lesions which can be performed by localizing the WCE in the GI tract. In this paper, we propose ultra-wideband (UWB) path loss-based WCE localization and compute the Cramer–Rao lower bound (CRLB) to evaluate the accuracy bounds of localization in the small intestine. First, we propose the estimation of smoothed path loss by minimizing the path loss deviations caused by shadow fading effects of body tissues. Then, the estimated path loss is used to estimate the degree of path loss and to compute the weight of the sensor's positions. Finally, we propose the smoothed path loss degree-based weighted centroid localization (SPLD-WCL) algorithm to estimate the location of the WCE. We simulate the proposed SPLD-WCL algorithm and verify the accuracy by comparing it to the computed CRLB. The proposed SPLD-WCL localization algorithm shows a significantly high accuracy of localization with a 6.83 mm root mean square error (RMSE) without any advanced knowledge of unknown parameters and bounds.

## 1. Introduction

Wireless capsule endoscopy diagnoses the abnormalities in the gastrointestinal tract by sending images of the GI tract to an external device by wireless communication. For diagnosis, the physicians require to know the location of the WCE while capturing the image of the abnormalities. There are several WCE localization techniques based on magnetic field strength [1–3], radio frequency (RF) [4], or hybrid methods [5, 6]. The received signal strength indicator (RSSI)-based WCE localization techniques are generally based on triangulation or trilateration-based algorithms [4]. The authors of reference [7] propose triangulation-based 2*D* positioning of the *in vivo* RF signal where the signal strength is measured using a wearable antenna array for multiple points of the capsule to estimate the distance. The reported average error in [8] is 37.7 mm. In [9], the authors exploit spatial sparsity to estimate the position of the emitter using the tissue-adaptive method without estimating the time of arrival (ToA) or path loss. The authors of reference [9] use the convex optimization theory and *l*_1_-norm minimization to estimate the position and report less than 7.5 mm RMSE with a perfectly known tissue structure and less than 8.8 mm with an approximately known tissue structure with some levels of uncertainties.

The localization accuracy of the above traditional RSSI-based methods is influenced by the hostile RF signal propagation due to the nonhomogeneous tissue properties of the human body. Therefore, new approaches that are robust to channel estimation errors are proposed. In [10, 11], the authors propose RSSI-based maximum likelihood (ML) localization using finite impulse response (FIR) and particle filter-based tracking to find the transition model of the capsule. The authors of reference [11] reported 15 mm RMSE using the FIR filter and 7 mm RMSE using the particle filter-based approach. In [12], the authors use the RSSI-based weighted centroid localization (WCL) approach for capsule localization and reported 24.53 mm RMSE.

International regulatory organizations such as Federal Communications Commission (FCC) [13] recommend medical implant communication service (MICS) band for implant applications which is used in the above-proposed methods of localization [4, 7–12, 14]. However, high-data-rate communication with impulse radio ultra-wideband (IR-UWB) transceivers is also suitable and safe for implantable devices, and it does not interfere much with other radio devices [15]. Short-range, wireless communication using UWB frequency bands is also defined in the IEEE standard 802.15.6 in the vicinity of, or inside, a human body [13]. The IEEE standard UWB signal propagation models for implantable devices are presented in [13, 16, 17]. Several UWB-based WCE localization algorithms are available in the literature [18–20].

The authors of reference [18] propose UWB RSS-based capsule endoscopy localization using compressive sensing and the variable noise level (VNL) Kalman filter. The localization error is 35–60 mm based on the frequency of operation as reported in [18]. In [19], the authors propose UWB 2 × 2 MIMO diversity to estimate the path loss and position-bounded calibrated WCL to localize the capsule in the small intestine. The reported localization accuracy of the MIMO-based approach in [19] is 5.14 mm RMSE using position bounds, whereas it is 7.49 mm without position bounds. However, due to the size and space limitation, higher-order diversity antennas are difficult to be equipped in the capsule, and only 3-dB diversity gain is recommended in [21] for space diversity due to the high correlation among different on-body receiver locations. In [20], the authors propose ML estimation for UWB path loss estimation and propose WCL-based localization using position bounds and path loss bounded weight of the sensor receivers. In [20], the reported RMSE error is 6.2 mm for capsule localization in the small intestine using position bounds and 8.14 mm RMSE without using the position bounds. However in [19, 20], the authors simulate the proposed capsule localization using the statistical description of UWB propagation through the human chest [16] which is not a suitable scenario for localization in the small intestine. In [19], a calibration coefficient is used which requires prior knowledge of the dimension of the small intestine. Again, for position estimation in both [19, 20], position bounds are applied that are computed using the dimension of the small intestine which is practically not feasible. Most of the above-reported works are on developing RSSI-based capsule localization algorithms only. In [22], the authors calculate the accuracy bounds of the RF-based triangulation method for capsule localization using a log-normal channel model of the MICS band. However, no research work is reported in the literature on the accuracy bound of UWB-based WCE localization which can be used as the benchmark to compare the accuracy. Further, in the previous works [4, 7–12, 18–20], the statistical signal propagation using the MICS or UWB frequency band is modeled using the finite-difference time-domain (FDTD), the finite integration technique (FIT), or electromagnetic field simulators, where the signal reflections, blood flow, respiration, body movements, antenna alignment, etc. related factors are not considered.

In this paper, we propose a novel method of localization of the WCE using UWB path loss. We also derive and compute the CRLB as the benchmark of the accuracy of the proposed WCE localization in the small intestine. To generate the path loss and to compute the CRLB, we model a small intestine trajectory and map the coordinate values for varying locations of the WCE in the small intestine. Then, we use the distance between the mapped positions of the WCE and the reference positions of the sensor receivers to generate the UWB path loss using the statistics of the UWB path loss model extracted in [17] considering in-body to on-body *in-vivo* measurements scenario. Then, the CRLB is computed using the generated UWB path loss and the proposed scenario of WCE localization. We also propose a novel method of WCE localization using UWB path loss-based weighted centroid localization. Since the UWB path loss is highly deviated by the shadowing effects caused by the nonhomogeneous tissue properties of the human body, we propose the smoothed path loss estimation methods to mitigate the effect of path loss deviations on the accuracy of localization. We estimate the smoothed path loss by finding the best-fitted path loss of the neighboring location points followed by an averaging method. The path loss exponents of the best-fitted path loss are estimated by using linear least square regression of the scattered path loss of the neighboring location points. We also estimate the degree of the path loss using the standard deviation of the scattered path loss and the estimated smoothed path loss. Then, the smoothed path loss is raised to the degree to estimate the weight of the reference sensor receiver's positions. Finally, the position of the WCE is estimated by finding the weighted centroid of the reference sensor receiver's positions. We evaluate the impact of path loss deviations and the impact of the number of sensor receivers on the accuracy of localization. The proposed WCE localization algorithm outperforms the other state-of-the-art works in the literature without any prior knowledge of unknown parameters and position bounds. It can localize the capsule with an accuracy of 6.83 mm RMSE which is very close to the computed CRLB.

## 2. Localization System Architecture

We propose a WCE localization system, where the WCE is localized using a body-surrounded 3D sensor array of multiple sensor receivers as shown in Figure 1. The 3D sensor array is placed around the abdominal region of the human body. Here, we consider the transmitter (Tx) to be equipped with the WCE and the sensor receivers (Rx) to be equipped with miniaturized impulse radio (IR) UWB transceivers [15] suitable for the wireless body area network (WBAN).

In our proposed localization approach, the Tx inside the WCE travels through *M* possible target positions in the small intestine and transmits the UWB signal. The signal is received by the *N* sensor receivers of the sensor array. The RSSI is measured by the *N* sensor receivers for varying location points of the WCE transmitter in the small intestine. The scattered path loss is calculated using the transmitted power and the received signal strength. Since the path loss is highly deviated due to the body tissue properties of the human body, the smoothed path loss is estimated using our proposed method. Then, the degree of path loss is estimated using our proposed method. As the path loss attenuates with the distance, we consider the path loss as a measure of the Tx-Rx separation distance and compute the weight of the sensor receiver's position using the estimated path loss raised to the degree. Finally, the coordinate position of the WCE is estimated using weighted centroid localization by finding the weighted centroid of the reference positions of the sensor receivers.

## 3. Path Loss Model

In our proposed localization approach, the UWB signal between the capsule transmitter and the body-surrounded sensor receivers is scattered due to the different material dielectric properties of human body layers along the propagation path. Using the practical scenario, the scattered path loss can be found using the measured RSSI and transmitted power as follows:

(1) $$\begin{array}{c} L_{i}\left(dB\right)=P_{T}\left(dB\;m\right)-RSSI\left(dB\;m\right)\text{,} \end{array}$$

where, *L*_*i*_ is the scattered path loss and *P*_*T*_ is the transmitted power. The scattered UWB path loss is represented as follows:

(2) $$\begin{array}{c} L_{i}=\alpha \left(\frac{r_{i}}{r_{0}}\right)+L\left(r_{0}\right)+X\left(\mu ,\sigma_{L}^{2}\right)\text{,} \end{array}$$

where *α*, *r*_*i*_, *r*_0_, and *L*(*r*_0_) denote the fitting constant, separation distance between the capsule transmitter (Tx) and the *i*^th^ sensor receiver (Rx), reference Tx-Rx distance at 1cm, and the path loss in *d*B at reference distance *r*_0_, respectively. The statistical distribution *X*(*μ*, *σ*_*L*_^2^) of the shadowing term follows a Gaussian distribution model with mean *μ* and standard deviation of *σ*_*L*_.

Short-range, wireless communication using UWB frequency inside a human body is specified in the IEEE standard 802.15.6 and characterized by very low power consumption, the smaller size of the antennas, and a higher data rate [13, 17]. In [17], the statistics of the UWB signal propagation using a frequency band covering from 3.1 to 6 GHz are extracted using in vivo measurements, where the on-body receiving antennas are located on the abdomen and the in-body positions are located in the small bowel or the colon. The extracted statistics of the path loss are specified in Table 1. We generate the scattered UWB path loss using equation (2) by replacing the value of *r*_*i*_ and the statistics as available in Table 1. The Tx-Rx separation distance *r*_*i*_ is found for each of the traveling positions of WCE in the small intestine as follows:

(3) $$\begin{array}{c} r_{i}=\sqrt{{\left(x_{r}-x_{i}\right)}^{2}+{\left(y_{r}-y_{i}\right)}^{2}+{\left(z_{r}-z_{i}\right)}^{2}}\text{,} \end{array}$$

where, (*x*_*r*_, *y*_*r*_, *z*_*r*_) are the coordinates of the real position of the capsule transmitter and (*x*_*i*_, *y*_*i*_, *z*_*i*_) are the coordinates of the reference position of the *i*^th^ sensor receiver.

## 4. CRLB on the Localization Accuracy

In this section, we analyze and compute the accuracy limit of WCE localization in the small intestine by finding the Cramer–Rao lower bound which provides a benchmark against the accuracy of an unbiased estimator [23]. Therefore, we derive the CRLB as the accuracy bounds of WCE localization by determining the relationship between the path loss estimation error and the location estimation error. This is because the accuracy of WCE localization is mostly influenced by the path loss estimation error. The path loss estimation error occurs due to the scattering of the path loss caused by the nonhomogeneous tissue properties of the human body.

The scattered path loss is represented as equation (2), where *X*(*μ*, *σ*_*L*_^2^) is the scattered shadowing term with mean *μ* and standard deviation of *σ*_*L*_. Thus, the best-fitted mean path loss excluding the scattering term can be expressed as follows:

(4) $$\begin{array}{c} \bar{L}\left(r_{i}\right)=\alpha \left(\frac{r_{i}}{r_{0}}\right)+L\left(r_{0}\right)\text{,} \end{array}$$

and the standard deviation of path loss, *σ*_*L*_, can be given as follows:

(5) $$\begin{array}{c} \sigma_{L}=\sqrt{\frac{1}{N}\overset{N}{\underset{i=1}{\sum }}{\left(L_{i}-\bar{L}\left(r_{i}\right)\right)}^{2}}\text{,} \end{array}$$

where *N* is the total number of sensor receivers. In the following subsections, we estimate the CRLB on the variance of path loss to relate it to the CRLB of the localization error.

### 4.1. CRLB on the Variance of Path Loss

The probability density function (PDF) of the path loss with random white Gaussian noise (WGN) shows Gaussian distribution with mean $\bar{L}\left(r_{i}\right)$ and standard deviation *σ*_*L*_ as shown in the following:

(6) $$\begin{array}{c} p\left(L_{i};\bar{L}\left(r_{i}\right)\right)=\frac{1}{{\left(2\pi \sigma_{L}^{2}\right)}^{N/2}}\exp\;\left[-\frac{1}{2\sigma_{L}^{2}}\overset{N}{\underset{i=1}{\sum }}{\left(L_{i}-\bar{L}\left(r_{i}\right)\right)}^{2}\right]\text{.} \end{array}$$

The Cramer–Rao lower bound (CRLB) on the variance of the path loss estimator must satisfy the following equation:

(7) $$\begin{array}{c} var\left(\bar{L}\left(r_{i}\right)\right)>=\frac{1}{-E\left[d^{2}\;\ln\;\left[p\left(L_{i};\bar{L}\left(r_{i}\right)\right)\right]/d{\bar{L}}^{2}\right]}\text{.} \end{array}$$

Differentiating the logarithm of equation (6) once with respect to best-fitted mean path loss $\left(\bar{L}\right)$, we get the following equation:

(8) $$\begin{array}{c} \frac{d\;\ln\;\left[p\left(L_{i};\bar{L}\left(r_{i}\right)\right)\right]}{d\bar{L}}=\frac{d}{d\bar{L}}\left[-\ln\left({\left(2\pi \sigma_{L}^{2}\right)}^{N/2}-\frac{1}{2\sigma_{L}^{2}}\overset{N}{\underset{i=1}{\sum }}{\left(L_{i}-\bar{L}\left(r_{i}\right)\right)}^{2}\right)\right]\\ =\frac{1}{\sigma_{L}^{2}}\overset{N}{\underset{i=1}{\sum }}\left(L_{i}-\bar{L}\left(r_{i}\right)\right)\text{.} \end{array}$$

The expected path loss $\bar{L}\left(r_{i}\right)$ can be achieved by equating equation (8) to zero. Differentiating equation (8) results in the following equation:

(9) $$\begin{array}{c} \frac{d^{2}\;\ln\;\left[p\left(L_{i};\bar{L}\left(r_{i}\right)\right)\right]}{d{\bar{L}}^{2}}=-\frac{N}{\sigma_{L}^{2}}\text{.} \end{array}$$

Thus, CRLB on the variance of path loss is obtained as follows:

(10) $$\begin{array}{c} var\left(\bar{L}\left(r_{i}\right)\right)>=\frac{\sigma_{L}^{2}}{N}\text{.} \end{array}$$

### 4.2. CRLB on the Variance of Localization

The PDF of path loss for an unknown location of the capsule can be expressed as follows:

(11) $$\begin{array}{c} p\left(L_{i};r_{i}\right)=\frac{1}{{\left(2\pi \sigma_{L}^{2}\right)}^{N/2}}\exp\;\left[-\frac{1}{2\sigma_{L}^{2}}\overset{N}{\underset{i=1}{\sum }}{\left(L_{i}-\bar{L}\left(r_{i}\right)\right)}^{2}\right]\text{,} \end{array}$$

where *r*_*i*_ is the distance between Tx-Rx, and it is a function of the 3*D* coordinate (*x*, *y*, *z*) positions of the capsule. The CRLB on the variance of the location estimator must satisfy the following equation:

(12) $$\begin{array}{c} var\left(r_{i}\right)>=\frac{1}{-E\left[d^{2}\;\ln\left(p\left(L_{i};r_{i}\right)\right)/dx^{2}dy^{2}dz^{2}\right]}\text{.} \end{array}$$

Differentiating the logarithm of equation (11) once with respect to *x*-*y*-*z* coordinate positions, we get the following equation:

(13) $$\begin{array}{c} \frac{d\;\ln\;\left[p\left(L_{i};r_{i}\right)\right]}{dx\;dy\;dz}=\frac{d}{dx\;dy\;dz}\left[-\ln\left({\left(2\pi \sigma_{L}^{2}\right)}^{N/2}-\frac{1}{2\sigma_{L}^{2}}\overset{N}{\underset{i=1}{\sum }}{\left(L_{i}-\bar{L}\left(r_{i}\right)\right)}^{2}\right)\right]\\ =\frac{1}{\sigma_{L}^{2}}\overset{N}{\underset{i=1}{\sum }}\left(L_{i}-\bar{L}\left(r_{i}\right)\right)\frac{d\bar{L}\left(r_{i}\right)}{dx\;dy\;dz}\text{.} \end{array}$$

Differentiating (13), we get thefollowing equation:

(14) $$\begin{array}{c} \frac{d^{2}\;\ln\;\left[p\left(L_{i};r_{i}\right)\right]}{dx^{2}dy^{2}dz^{2}}=-\frac{N}{\sigma_{L}^{2}}{\left[\frac{d\bar{L}\left(r_{i}\right)}{dx\;dy\;dz}\right]}^{2}\text{.} \end{array}$$

Thus, the CRLB on the variance of localization is obtained as follows:

(15) $$\begin{array}{c} var\left(r_{i}\right)>=\frac{\sigma_{L}^{2}}{N{\left(d\bar{L}\left(r_{i}\right)/dx\;dy\;dz\right)}^{2}}\text{.} \end{array}$$

To compute the CRLB, we differentiate the expected mean path loss $\bar{L}\left(r_{i}\right)$ in equation (4) with respect to *x*-*y*-*z* coordinates and get the following equation:

(16) $$\begin{array}{c} d\bar{L}\left(r_{i}\right)=\frac{\alpha }{2}\frac{r_{i}^{-1}}{r_{0}}\left[2\left(x-x_{i}\right)dx+2\left(y-y_{i}\right)dy+2\left(z-z_{i}\right)dz\right]\\ =\frac{\alpha }{r_{0}r_{i}}\left[\left(x-x_{i}\right)dx+\left(y-y_{i}\right)dy+\left(z-z_{i}\right)dz\right]\text{.} \end{array}$$

The equation (16) can be written in matrix form as follows:

(17) $$\begin{array}{c} \begin{array}{c} Hdr \end{array}\text{,} \end{array}$$

(18) $$\begin{array}{c} and\;we\;can\;write,{\left(\frac{d\bar{L}}{dr}\right)}^{2}=H^{\prime }H\text{,} \end{array}$$

(19) $$\begin{array}{c} where,\;d\bar{L}=\left(\begin{array}{c} d\bar{L}\left(r_{2}\right)\\ \vdots \\ d\bar{L}\left(r_{N}\right)\text{;} \end{array}\right),dr=\left(\begin{array}{c} dy\\ dz \end{array}\right)\;and \end{array}$$

Finally, replacing equations (18) and (15), the CRLB on the variance of localization is obtained as follows:

(20) $$\begin{array}{c} var\left(r\right)=\frac{\sigma_{L}^{2}}{N}\;{\left(H^{\prime }H\right)}^{-1}\begin{array}{cc} = & \left(\begin{array}{ccc} \sigma_{x}^{2} & \sigma_{xy}^{2} & \sigma_{zx}^{2}\\ \sigma_{xy}^{2} & \sigma_{y}^{2} & \sigma_{yz}^{2}\\ \sigma_{xz}^{2} & \sigma_{yz}^{2} & \sigma_{z}^{2} \end{array}\right). \end{array} \end{array}$$

Thus, we can compute the CRLB on the localization error as follows:

(21) $$\begin{array}{c} \sigma_{r}=\sqrt{\sigma_{x}^{2}+\sigma_{y}^{2}+\sigma_{z}^{2}}\text{.} \end{array}$$

For *M* possible positions of the capsule, the CRLB on the root mean square error (RMSE) of localization can be computed as follows:

(22) $$\begin{array}{c} CRLB_{RMSE}=\sqrt{\frac{\sum_{j=1}^{M}\left(\sigma_{x_{j}}^{2}+\sigma_{y_{j}}^{2}+\sigma_{z_{j}}^{2}\right)}{M}}\text{.} \end{array}$$

## 5. Proposed WCE Localization Algorithm

We propose a WCL-based localization algorithm to localize the three dimensional position of the WCE in the small intestine. WCL estimates the position of the implanted capsule by finding the weighted average of the sensor receivers' position as follows:

(23) $$\begin{array}{c} P\left(x_{e},y_{e},z_{e}\right)=\frac{\sum_{i=1}^{N}\left(W_{i}S_{i}\left(x_{i},y_{i},z_{i}\right)\right)}{\sum_{i=1}^{N}W_{i}}\text{,} \end{array}$$

where, *P*(*x*_*e*_, *y*_*e*_, *z*_*e*_) is the estimated *x*-*y*-*z* coordinate position of the capsule, *N* is the number of sensor receivers, *S*_*i*_(*x*_*i*_, *y*_*i*_, *z*_*i*_) is the reference *x*-*y*-*z* coordinate position of the *i*^th^ sensor receiver, and *W*_*i*_ is the weight of the reference position of the *i*^th^ sensor receiver which is inversely proportional to the distance of the sensor receivers from the capsule transmitter.

The detail methodologies of the proposed algorithm are shown in Algorithm 1 and explained in the following:

### 5.1. Path Loss Estimation

Path loss is estimated as a measure of Tx-Rx distance and to compute the weight of the reference positions of the sensor receivers. The propagation path loss is scattered due to the shadowing effect caused by the nonhomogeneous human tissue dielectric properties. To get an accurate estimate of the path loss, the scattering of the path loss is required to be minimized. The capsule travels *M* possible points through the small intestine. The best-fitted path loss of the adjacent traveling location points can be estimated as follows:

(24) $$\begin{array}{c} {\bar{L}}_{ik}=c_{1}k+c_{2}, \end{array}$$

where *k*=(*j* − *n*_*L*_) : (*j*+*n*_*R*_) is the range of *n*_*R*_+*n*_*L*_+1 adjacent location points of the capsule at *j*^th^ instant, *n*_*L*_ is the lower bound, *n*_*R*_ is the upper bound of the adjacent location points, and *c*_1_ and *c*_2_ are the path loss exponents. The path loss exponents are estimated by using linear least square regression of the scattered path loss measured at the adjacent location points of the capsule as follows:

(25) $$\begin{array}{c} C={\left(K^{T}K\right)}^{-1}K^{T}L\text{,} \end{array}$$

where **C** is a matrix of the path loss exponents, **L** is the matrix of the measured path loss of *n*_*R*_+*n*_*L*_+1 adjacent location points of the capsule, and **K** is the set of *n*_*R*_+*n*_*L*_+1 adjacent location points.

(26) $$\begin{array}{c} C=\left(\begin{array}{c} c_{1}\\ c_{2} \end{array}\right),L=\left(\begin{array}{c} L_{i\left(j-n_{L}\right)}\\ L_{i\left(j-n_{L+1}\right)}\\ \vdots \\ L_{i\left(j+n_{R-1}\right)}\\ L_{i\left(j+n_{R}\right)} \end{array}\right)and\;K=\left(\begin{array}{c} j-n_{L}\\ j-n_{L+1}\\ \vdots \\ j+n_{R-1}\\ j+n_{R} \end{array}\right)\text{.} \end{array}$$

Using the extracted path loss exponents *c*_1_ and *c*_2_, we can estimate the smoothed path loss, *PL*_*ij*_, between the *i*^th^ sensor receiver and *j*^*th*^ location point by averaging the best-fitted mean path loss of the adjacent location points as follows:

(27) $$\begin{array}{c} PL_{ij}=\frac{1}{\left(n_{R}+n_{L}+1\right)}\overset{j+n_{R}}{\underset{k=j-n_{L}}{\sum }}{\bar{L}}_{ik}=\frac{1}{\left(n_{R}+n_{L}+1\right)}\overset{j+n_{R}}{\underset{k=j-n_{L}}{\sum }}\left(c_{1}k+c_{2}\right). \end{array}$$

### 5.2. Weight Calculation

The weight of the reference position of the sensor receivers is inversely proportional to Tx-Rx distance. As the path loss is a measure of Tx-Rx distance, we can compute the weight using the estimated smoothed path loss and the estimated degree of path loss as follows:

(28) $$\begin{array}{c} W_{ij}=\frac{1}{PL_{ij}^{\gamma }}\text{,} \end{array}$$

where *γ* is the degree of path loss. *γ* is dependent on the propagation path loss caused by the shadowing environment. Thus, we can estimate the degree *γ* by finding the standard deviation of path loss (*σ*_*L*_) as follows:

(29) $$\begin{array}{c} \gamma =\sigma_{L}=\sqrt{\frac{1}{MN}\overset{N}{\underset{i=1}{\sum }}\overset{M}{\underset{j=1}{\sum }}{\left(L_{ij}-PL_{ij}\right)}^{2}}\text{,} \end{array}$$

where *M* is the number of location points, *N* is number of sensor receivers, and *L*_*ij*_ and *PL*_*ij*_ are the measured scattered path loss and the estimated smoothed path loss between the *i*^th^ sensor receiver and the *j*^th^ location position of the capsule, respectively.

### 5.3. Position Estimation

Finally, we estimate the 3D position of the capsule using WCL. We put the calculated weight of the sensor receiver's position in equation (23) and estimate the *j*^th^ instant position of the capsule as follows:

(30) $$\begin{array}{c} P_{j}\left(x_{e},y_{e},z_{e}\right)=\frac{\sum_{i=1}^{N}\left({1/PL_{ij}^{\gamma }S}_{i}\left(x_{i},y_{i},z_{i}\right)\right)}{\sum_{i=1}^{N}1/PL_{ij}^{\gamma }}\text{.} \end{array}$$

## 6. Performance Metrics

We apply the following three performance metrics to evaluate the accuracy of the proposed path loss estimation and position estimation methods.

### 6.1. Coefficient of Determination, *R*^2^

The coefficient of determination (*R*^2^) measures how well a statistical model predicts an outcome. The outcome is represented by the model's dependent variable. The lowest possible value of *R*^2^ is 0, and the highest possible value is 1. The better a model is at making predictions, the closer its *R*^2^ will be to 1. The formula of the coefficient of determination (*R*^2^) is as follows:

(31) $$\begin{array}{c} R^{2}=1-\frac{RSS}{TSS}\text{,} \end{array}$$

where RSS is the sum of squared residuals and TSS is the total sum of squares. We use *R*^2^ to verify the performance of the proposed path loss estimation and position estimation methods. For the path loss estimation method, we calculate the coefficient of determination of path loss, *R*_*pl*_^2^, as follows:

(32) $$\begin{array}{c} R_{pl}^{2}=1-\frac{\sum {\left(Original\;path\;loss-Estimated\;path\;loss\right)}^{2}}{\sum {\left(Original\;path\;loss-Mean\;of\;original\;path\;loss\right)}^{2}}\text{.} \end{array}$$

For our proposed position estimation, we calculate the coefficient of determination of position, *R*_pos_^2^, as follows:

(33) $$\begin{array}{c} R_{pos}^{2}=1-\frac{\sum {\left(Original\;position-Estimated\;position\right)}^{2}}{\sum {\left(Original\;position-Mean\;of\;original\;positions\right)}^{2}}\text{.} \end{array}$$

### 6.2. Localization Error (LE)

The localization error is a performance metric that is simply measured by the difference between estimated and real positions as follows:

(34) $$\begin{array}{c} LE=\sqrt{{\left(x_{r}-x_{e}\right)}^{2}+{\left(y_{r}-y_{e}\right)}^{2}+{\left(z_{r}-z_{e}\right)}^{2}}\text{,} \end{array}$$

where (*x*_*r*_, *y*_*r*_, *z*_*r*_) are the coordinates of the real positions and (*x*_*e*_, *y*_*e*_, *z*_*e*_) are the coordinates of the estimated positions. The LE is compared to the computed CRLB of the LE as a benchmark to verify the accuracy of localization.

### 6.3. Root Mean Square Error (RMSE)

The RMSE is a performance metric which is computed as follows:

(35) $$\begin{array}{c} RMSE=\sqrt{\frac{\sum_{j=1}^{M}\left[{\left(x_{r_{j}}-x_{e_{j}}\right)}^{2}+{\left(y_{r_{j}}-y_{e_{j}}\right)}^{2}+{\left(z_{r_{j}}-z_{e_{j}}\right)}^{2}\right]}{M}}\text{,} \end{array}$$

where *M* is the total number of possible positions traveled by the capsule, (*x*_*r*_*j*__, *y*_*r*_*j*__, *z*_*r*_*j*__) are the coordinates of the *j*^th^ real position of the capsule, and (*x*_*e*_*j*__, *y*_*e*_*j*__, *z*_*e*_*j*__) are the coordinates of the *j*^th^ estimated position of the capsule. The RMSE is compared to the computed CRLB of the RMSE as a benchmark to verify the accuracy of localization.

## 7. Simulation and Results

We simulate the proposed localization algorithm using a 3D simulation platform developed in MATLAB as shown in Figure 2. The simulation platform includes 48 sensor receivers (Rx) placed at the corner points of a 3*D* cubic sensor array of 200 mm × 200 mm × 200 mm dimension. The 48 sensor receivers are placed as a cluster of six (06) sensor receivers at 8 corner points of the sensor array. The distance between the clustered sensor receivers is kept at 30 mm to reduce frequency interference. The simulation platform also includes a 2443 mm long small intestine trajectory model. The traveling path in the small intestine is mapped with 2443 coordinate positions of the capsule transmitter (Tx) in 1 mm resolution. The communication between the capsule transmitter (Tx) and the sensor receivers (Rx) is modeled using UWB signal propagation with 8 *dB*_*m*_ output power and highly deviated path loss due to the different material dielectric properties of human body layers. The simulation parameters are summarized in Table 2.

To evaluate the performance of the proposed localization algorithm, we use three performance metrics, *R*_pos_^2^, the LE and the RMSE, as shown in equations (33), (34), and (35), respectively. To compare the performance to a benchmark accuracy, we compute the CRLB on the variance of localization as shown in equation (20). It is apparent from equation (20) that the performance is dependent on the standard deviation of path loss *σ*_*L*_ and the Tx-Rx separation distance. As we know that for our proposed localization approach, the path loss is highly deviated due to the material properties of the human body layers. Therefore, to generate the scattered path loss between the Tx-Rx, we use the statistical path loss parameters as specified in Table 1 that are extracted in [17] for ingestible devices using the in-body to on-body in vivo measurement scenario. Then, we generate the scattered path loss and best-fitted mean path loss using equations (2) and (4), respectively, by replacing the value of Tx-Rx separation distance *r*_*i*_ and the path loss statistics as available in Table 1. The distance *r*_*i*_ between the reference coordinate positions of the sensor receivers and all the mapped 2443 traveling positions of the capsule are calculated using equation (3).  Figure 3 illustrates how the path loss varies with the Tx-Rx separation distance and how the path loss is scattered around the best-fitted path loss due to the standard deviation of path loss *σ*_*L*_. The path loss deviation *σ*_*L*_ and the channel response **H** are calculated using equations (5) and (19) for different number of sensor receivers and replaced in equation (20) to compute the CRLB on the variance of localization. Finally, the CRLB on the LE and the RMSE are computed using equation (21) and (22), respectively.  Figure 4 shows the CRLB on the LE for all positions as a function of the standard deviation of path loss, *σ*_*L*_. It is observed in Figure 4 that the CRLB on the LE increases with path loss deviation *σ*_*L*_.

To minimize the deviation in the scattered path loss, we estimate the smoothed path loss using our proposed method using equation (27). The path loss exponents *c*_1_ and *c*_2_ are estimated using LLS regression as shown in equation (26). The lower and upper bound of the adjacent location points were set to 11 to obtain optimal results. The performance of our proposed path loss estimation method is evaluated using the performance metric *R*_*pl*_^2^ as shown in equation (32). The *R*_*pl*_^2^ value using 8 sensor receivers is 0.9971 and using 48 sensor receivers is 0.9974, indicating a very high coefficient of determination at making predictions.

Next, we simulate the proposed smoothed path loss degree-based WCL (SPLD-WCL) algorithm using 8–48 sensor receivers to estimate the position of the capsule traveling through the small intestine. Figure 2 shows the simulation results with 48 sensor receivers and illustrates the real and estimated positions of 2443 simulated positions of the capsule in the small intestine trajectory. The performance is evaluated using the *R*_pos_^2^, the LE, and the RMSE.  Table 3 summarizes the results obtained using different improvement steps of the algorithm. It is observed from the results in Table 3 that the *R*_pos_^2^ improves and the RMSE reduces significantly by applying different improvement steps of the proposed algorithm.  Figure 5 illustrates the localization error of all simulated positions by applying different improvement steps of the proposed algorithm. It is apparent from Table 3 and Figure 5 that a major improvement is obtained by applying the improvement steps, especially by applying path loss smoothing and by raising the path loss to the estimated degree *γ*. It is also observed that the accuracy is improved by raising the degree of both the scattered path loss and the smoothed path loss.  Figure 5 and Table 3 also compare the accuracy to the computed CRLB. It is observed that the localization error and the RMSE of the proposed methods are very close to the computed CRLB.

We analyze the impact of the sensor receivers on the accuracy of the localization by varying the number of sensor receivers from 8 to 48. In our proposed approach of localization using WCL, the WCE is localized by finding the weighted centroid of the sensor receivers' positions. Therefore, at least 8 sensor receivers are required to be placed at the 8 corner points of the 3D cubical array to localize the capsule traveling through the central locations of the cube by finding the weighted centroid. It is observed in Table 3 that using four (04) sensor receivers, we obtain a negative *R*_pos_^2^ value. Thus, a minimum of 8 receivers are required for 3D localization of the WCE using WCL. The cumulative distribution of the localization error (LE) for an increasing number of sensor receivers is demonstrated in Figure 6. It is observed that for 2443 simulated positions, 80% of localization error remains below 12 mm by using 8 sensor receivers, whereas by using 48 sensor receivers, 80% of the localization errors remain below 10 mm.  Figure 7 illustrates the RMSE accuracy of the proposed SPLD-WCL for an increasing number of sensor receivers and compares it to the computed CRLB. It is observed in Figure 7 that the RMSE of the proposed SPLD-WCL algorithm and the CRLB decrease with the increasing number of sensor receivers. The computed CRLB on the RMSE is 3.96 mm and 0.664 mm using 8 and 48 sensor receivers, respectively. For 2443 simulated positions of the capsule, the RMSE of localization using the proposed SPLD-WCL localization algorithm is 8.7 mm and 6.83 mm using 8 and 48 sensor receivers, respectively.

Table 4 compares the methods and the obtained localization accuracy of the proposed SPLD-WCL algorithm to other works in the literature. As we can see from the comparison in Table 4, the proposed localization algorithm shows significantly high localization accuracy using 8 to 48 sensor receivers using the in-vivo UWB channel model as compared to the state-of-the-art methods of other works in the literature by applying the proposed methods of smoothed path loss estimation, path loss-based degree estimation, and the WCL. Thus, it may be concluded that the proposed SPLD-WCL localization algorithm outperforms the literature without any prior knowledge of unknown parameters, distance, or channel statistics with a significantly high accuracy close to the benchmark CRLB.

## 8. Conclusion

In this paper, we have proposed WCE localization in the small intestine using the SPLD-WCL algorithm using the UWB signal propagation between the capsule transmitter and sensor receivers of the body-surrounded sensor array. We have also found the CRLB as the benchmark of localization accuracy using the UWB signal propagation model. The performance of the proposed algorithm has been evaluated using the performance metrics, *R*^2^, the LE, and the RMSE. For the simulation, we have modeled a small intestine trajectory mapped with 2443 target positions of the WCE in 1 mm resolution. Then, we have generated the path loss using the UWB path loss statistics and the coordinate positions of the WCE in the small intestine trajectory model and the sensor receivers in the proposed localization scenario. Next, we have computed the CRLB on the LE and the RMSE using the generated path loss for the proposed localization scenario. The computed CRLB on the RMSE is 3.96 mm and 0.664 mm using 8 and 48 sensor receivers, respectively. To develop the proposed localization algorithm, we have proposed smoothed path loss estimation to minimize the effect of the path loss deviation on the localization accuracy. We have also proposed a method of determining the degree of the path loss using the standard deviation of the scattered path loss and the smoothed path loss which does not require knowledge of any unknown parameters. Then, we have computed the weight of the sensor receivers using the estimated path loss raised to the degree and found the position of WCE using weighted centroid localization. We have simulated the proposed localization algorithm to localize the WCE at 2443 target positions in the small intestine. The proposed methods show significantly high accuracy in path loss estimation and localization of the WCE in the small intestine. The accuracy of the path loss estimation methods in terms of *R*_*pl*_^2^ is 0.9971 and 0.9974 using 8 and 48 sensor receivers, respectively, indicating a very high level of significance in making predictions. We have also analyzed the impact of the number of sensor receivers and the path loss variance on localization accuracy. We have seen that the accuracy of localization improves by increasing the number of sensor receivers. It is also found that the accuracy of localization improves significantly by applying path loss smoothing and the degree of path loss. The measured coefficient of determination of the positions, *R*_pos_^2^, is 0.9901 which indicates a significantly high level of estimation. The simulation results show that the RMSE of the proposed localization algorithm is 8.7 mm and 6.83 mm using 8 and 48 sensor receivers, respectively, which is very close to the benchmark CRLB. Thus, it may be concluded that the proposed SPLD-WCL localization algorithm can obtain significantly high accuracy as compared to the state-of-the-art works in the literature without any prior knowledge of distances, bounds, and any unknown parameters.

## Figures and Tables

**Figure 1:** The system architecture of WCE localization.

**Figure 2:** The 3D simulation platform showing 2443 real and estimated trajectory positions of the capsule and the sensor receivers.

**Figure 3:** Path loss as a function of distance.

**Figure 4:** CRLB on the LE as a function of the standard deviation of path loss *σ*_*L*_ (considering 2443 simulated positions).

**Figure 5:** The localization error (LE) of 2443 simulated positions.

**Figure 6:** Cumulative distribution of the localization error.

**Figure 7:** The RMSE of localization as a function of number of sensor receivers.

**Algorithm 1:** UWB smoothed path loss degree-based WCL (SPLD-WCL).

**Table 1:** UWB path loss parameters for ingestible devices [17].

Scenario	*L*(*r*_0_)	*r*_0_	*α*	*μ*	*σ*_*L*_
In-body to on-body in vivo measurements	41.5635 *d*B	1cm	4.337	0	4.6007

**Table 2:** Simulation parameters.

Simulation parameters	Value
Frequency band	[3.1, 6] GHz
Dimension of the sensor array	200 × 200 × 200 mm
Number of sensor receivers, *N*	8–48
Spacing between the corner point sensors	30 mm
Length of the small intestine trajectory	2443 mm
Resolution of the mapped positions	1 mm
Dimension of the mapped positions	120 × 70 × 120 mm
Number of simulated positions, *M*	2443
Lower bound of adjacent points, *n*_*L*_	11
Upper bound of adjacent points, *n*_*R*_	11
Path loss at reference distance, *L*(*r*_0_)	41.5635
Fitting constant of path loss, *α*	4.337
Standard deviation of path loss, *σ*_*L*_	4.6007

**Table 3:** Accuracy of localization by applying different improvement steps.

Algorithm	Path loss	Degree of path loss	Weight basis	Sensor receivers	Positioning	*R*_pos_^2^	RMSE	CRLB
Scattered path loss-based WCL (SCPL-WCL)	Scattered	No degree	Scattered path loss	4	WCL	−1.95	119.8	8.77
SCPL-WCL	Scattered	No degree	Scattered path loss	8	WCL	0.319	57.54	3.96
SCPL-WCL	Scattered	No degree	Scattered path loss	48	WCL	0.316	57.67	0.664
Smoothed path loss-based WCL (SPL-WCL)	Estimated smoothed path loss	No degree	Smoothed path loss	8	WCL	0.319	57.56	3.96
SPL-WCL	Estimated smoothed path loss	No degree	Smoothed path loss	48	WCL	0.314	57.74	0.664
Scattered path loss degree-based WCL (SCPLD-WCL)	Scattered	Estimated degree	Scattered path loss raised to the degree	8	WCL	0.955	14.99	3.96
SCPLD-WCL	Scattered	Estimated degree	Scattered path loss raised to the degree	48	WCL	0.985	8.51	0.664
Smoothed path loss degree-based WCL (SPLD-WCL)	Estimated smoothed path loss	Estimated degree	Smoothed path loss raised to the degree	8	WCL	0.9837	8.7	3.96
SPLD-WCL	Estimated smoothed path loss	Estimated degree	Smoothed path loss raised to the degree	48	WCL	0.9901	6.83	0.664

**Table 4:** Comparison of the proposed SPLD-WCL algorithm to other works in the literature.

Localization method	Band	RMSE (mm)	No. of sensors	Dimension	*In vitro*or *in vivo* measurements
*Hybrid methods*					
Hybrid localization using vision and RF [5]	MICS	23	16	3*D*	Partially - image dataset from pillcam
Fusion based hybrid localization using vision and IMU sensors [6]	MICS	9.5	NO	3*D*	Yes - *in vitro* validation

*TOA and RSSI base*d					
TOA, path loss, and spatial sparsity-based convex optimization and *l*_1_-norm minimization [9]	MICS	8.0	16	2*D*	No - implant to the body surface model using electromagnetic field simulation

*RSSI based*					
RSSI based triangulation [24]	MICS	34	64	3*D*	No - implant to the body surface model using electromagnetic field simulation
Nonparametric path loss-based WCL [12]	MICS	24.53	64	3*D*	No - implant to the body surface model using electromagnetic field simulation
RSSI-based ML localization using the particle filter [11]	MICS	7.0	8	3*D*	No - FDTD simulation in the small intestine
RSSI-based compressive sensing and VNL Kalman filter [18]	UWB	35	24	2*D*	No - field simulation based
GWA filter and MIMO-based path loss estimation and position-bounded calibrated WCL [19]	UWB	8.24	56	3*D*	No - FIT simulation of human torso with electrical field probes inside the chest
		7.49			
ML estimated path loss-bounded WCL [20]	UWB	8.14	56	3*D*	No - FIT simulation of human torso with electrical field probes inside the chest
Proposed SPLD-WCL	UWB	8.7	8	3*D*	Yes - in-body to on-body *in vivo* measurements
		6.83	48		

## Data Availability

The dataset used to support the findings of this study is available from the corresponding author upon request.

## References

[1] Shao G., Tang Y., Tang L., Dai Q., Guo Y.-X. (2019). A novel passive magnetic localization wearable system for wireless capsule endoscopy. *IEEE Sensors Journal*.

[2] Sadeghi Boroujeni P., Pishkenari H. N., Moradi H., Vossoughi G. (2021). Model-aided real-time localization and parameter identification of a magnetic endoscopic capsule using extended kalman filter. *IEEE Sensors Journal*.

[3] Guo Y., Shao G. (2021). Wireless localization for a capsule endoscopy: techniques and solutions. *Antenna and Sensor Technologies in Modern Medical Applications*.

[4] Peter B., Machaj J. (2013). A novel enhanced positioning trilateration algorithm implemented for medical implant in-body localization. *International Journal of Antennas and Propagation*.

[5] Bao G., Pahlavan K., Mi L. (2015). Hybrid localization of microrobotic endoscopic capsule inside small intestine by data fusion of vision and RF sensors. *IEEE Sensors Journal*.

[6] Vedaei S. S., Wahid K. A. (2021). A localization method for wireless capsule endoscopy using side wall cameras and IMU sensor. *Scientific Reports*.

[7] Glukhovsky A., Frisch M., Levy D. (2002). Array system and method for locating an in vivo signal source.

[8] Fischer D., Schreiber R., Levi D., Eliakim R. (2004). Capsule endoscopy: the localization system. *Gastrointestinal Endoscopy Clinics of North America*.

[9] Pourhomayoun M., Jin Z., Fowler M. L. (2014). Accurate localization of in-body medical implants based on spatial sparsity. *IEEE Transactions on Biomedical Engineering*.

[10] Anzai D., Aoyama S., Wang J. (2012). Performance evaluation on RSSI-based localization for capsule endoscopy systems with 400MHz MICS band signals. *IEICE - Transactions on Communications*.

[11] Ito T., Anzai D., Wang J. (2014). Performance evaluation on RSSI-based wireless capsule endoscope location tracking with particle filter. *IEICE - Transactions on Communications*.

[12] Hany U., Akter L. (2018). Non-parametric method of path loss estimation for endoscopic capsule localization. *International Journal of Wireless Information Networks*.

[13] Chavez-Santiago R., Sayrafian-Pour K., Khaleghi A. (2013). Propagation models for IEEE 802.15. 6 standardization of implant communication in body area networks. *IEEE Communications Magazine*.

[14] Than T. D., Alici G., Zhou H., Li W. (2012). A review of localization systems for robotic endoscopic capsules. *IEEE Transactions on Biomedical Engineering*.

[15] Khaleghi A., Chávez-Santiago R., Balasingham I. (2010). Ultra-wideband pulse-based data communications for medical implants. *IET Communications*.

[16] Ali Khaleghi R. C., Santiago B. I., Chávez-Santiago R. (2011). Ultra-wideband statistical propagation channel model for implant sensors in the human chest. *IET Microwaves, Antennas & Propagation*.

[17] Perez-Simbor S., Andreu C., Garcia-Pardo C., Frasson M., Cardona N. (2019). UWB path loss models for ingestible devices. *IEEE Transactions on Antennas and Propagation*.

[18] Bjørnevik A. S. (2015). Localization and tracking of intestinal paths for wireless capsule endoscopy.

[19] Hany U., Akter L. (2017). Non-parametric approach of video capsule endoscope localization using suboptimal method of position bounded CWCL. *IEEE Sensors Journal*.

[20] Hany U., Akter L. (2018). Non-parametric approach using ML estimated path loss bounded WCL for video capsule endoscope localization. *IEEE Sensors Journal*.

[21] Shi J., Wang J. Channel characterization and diversity feasibility for in-body to on-body communication using low-band UWB signals.

[22] Wang Y., Fu R., Ye Y., Khan U., Pahlavan K. Performance bounds for RF positioning of endoscopy camera capsules.

[23] Kay S. M. (1993). *Fundamentals of Statistical Signal Processing: Estimation Theory*.

[24] Ye Y., Swar P., Pahlavan K., Ghaboosi K. (2012). Accuracy of RSS-based RF localization in multi-capsule endoscopy. *International Journal of Wireless Information Networks*.

